# Creating Sustainable Cultural Industries: The Perspective of Artificial Intelligence and Global Value Chain

**DOI:** 10.1155/2022/6768388

**Published:** 2022-08-22

**Authors:** Yutong Liu, Peiyi Song

**Affiliations:** School of Economics and Management, Communication University of China, Beijing 100024, China

## Abstract

In the era of artificial intelligence (AI), cultural industries have introduced new development opportunities, and their global value chain (GVC) position is receiving more attention. This study uses panel data from global cross-borders from 56 countries (regions) as the research sample to empirically analyze the impact of AI on improving the GVC position of cultural industries using the double fixed effects regression model and examines the heterogeneity effect. The results confirm that there is a significant positive correlation between AI and the GVC position of cultural industries. The mechanism test shows that AI impacts the division of labor position in the GVC of cultural industries mainly through technological innovation and the industrial structure. Heterogeneity analysis shows that AI has a significant effect on promoting the cultural industry's GVC position in high-income countries (regions) but it has no significant effect on low- and middle-income countries (regions). The results of this study can provide a useful reference for improving the division of labor positions in the GVC and better promoting the development of cultural industries.

## 1. Introduction

In the era of the digital economy, a new round of scientific and technological revolutions represented by AI is leading to the transformation of social productivity and the reconstruction of the GVC worldwide. At present, the world's major developed countries have begun to strategically deploy AI technology development at the national level, and AI has become a new competitive focus among major countries. With the rise of new technologies such as cloud computing, the Internet of Things, and big data, the development of AI has entered a new stage and is leading the transformation of cultural industries in many fields. The “culture + AI” industry continues to gain momentum. The deep integration of AI technologies such as deep learning, face recognition, intelligent search, and VR with cultural industries has created a new model of content production, dissemination, and consumption. Countries around the world are participating in a new round of global industrial competition with the help of the integrated development of cultural industries and AI technology. Therefore, the value chain of cultural industries is changing. It has become a general trend to introduce AI into content creation, development and production, marketing and promotion, communication and distribution, and consumer services in cultural industries.

Upgrades in AI technology will make it possible for the cultural industries to introduce a new development trend in technology and products, modes, and management. AI technology can promote the content creation of cultural products, improve the quality and efficiency of culture product development and production, transform the production mode of culture products on the production line as a whole, expand marketing channels and patterns, and integrate intelligence and personality. It has greatly enriched the means and content of communication and distribution, produced new experiential and scene-based consumption patterns, and promoted the innovation of cultural products. Furthermore, changes in the structure and organization of cultural industries have increased the size of cultural industries and expanded the layout area, and the integration of new and old industries has increased in both depth and breadth.

With the development of Internet technology and improvements in national infrastructure, more intermediate products are crossing borders multiple times, the segmentation of product production is being further refined, and the features of GVC are increasingly obvious. Countries specialize in the production of specific products in the value chain due to their resource endowment advantages, thus forming the “smile curve” of the international division of production. The high-quality development of cultural industries is an important aspect of high-quality economic development. In this context, it is of great significance to explore how AI technology affects the GVC division pattern of cultural industries to take advantage of strategic opportunities for AI development and realize high-quality economic development. Thus, this study uses panel data from 56 countries or regions from 2010 to 2018 to empirically analyze the impact of AI on the division position of labor in the GVC of cultural industries. Based on testing the robustness of the empirical results, the influence mechanisms of the impact of AI on improving the division position of labor in the GVC are discussed, and the influence of heterogeneity based on different stages of economic development is analyzed.

## 2. Literature Review

AI is a core issue in economic and social development. In 1940, Isaac Asimov proposed the “Three Principles of Robots,” aiming to protect human beings from the threat of robots [1]. After reviewing the literature, AI can be defined in the following two ways. First, at the technical level, AI is based on fuzzy logic, natural language processing technology, genetic algorithms, convolutional neural networks, adversarial generative networks, and artificial neural networks, and continues to develop [2–4]. Second, at the level of content, AI aims to simulate, extend, and expand human intelligence by using machines, the core of which is the learning of human thinking methods and processes by machines [5].

Research on AI and cultural industries focuses on three main aspects. First, it discusses the relationship between scientific and technological innovation and new forms of cultural industries and the role of science and technology in promoting the reform of cultural industries. This study indicates that the development of culture and technology promotes the repeated and orderly combination and extended use of cultural content to create new forms of products and advance their development to a higher level [6]. Second, the innovative application of AI technology in cultural industries and its impact on industrial development are discussed. Research indicates that the science of machine behavior is booming, using interdisciplinary research on machine behavior and related issues to explore how AI has evolved and what impact it may have on human society [7]. From the perspective of AI empowering cultural industries to improve quality and efficiency, related studies are carried out on the following aspects. At the macro-level, research shows that AI, big data, cloud computing, and Internet technology are highly compatible with the necessary conditions for the development of cultural industries, facilitating the accelerated integration of the cultural industry chain, the technique chain, and the innovation chain, thus realizing intelligent innovation and digital transformation [8, 9]. At the micro-level, with the aid of 5G technology and AI technology, diversified cultural equipment terminals augment the cultural experience of users [10]. Shahzad et al. [11] believed that smart TVs, mobile phones, smartwatches, and other devices as well as AR and VR technologies can better understand user psychology and provide experiential consumption of cultural services. In addition, from the perspective of the integrated development of old and new industries, such as the progress of the digital music industry, AI, machine learning, and big data make the coevolution of streaming music and live music possible [12]. Finally, in terms of AI's impact on economic growth, some scholars use the task-based model to examine the application of AI technology with the theoretical analysis framework of economics. Pioneering exploration has been conducted on how to achieve balanced economic growth under the application of AI technology, how the advancement of AI technology changes income factors of factor, and whether it leads to inequality [13].

Scholars have studied the division of labor in the GVC from different perspectives, including its measurement of the division of labor position in the value chain and influencing factors. Scholars have proposed a variety of indicators for measuring the division of labor in the GVC, such as the degree of upstream and downstream and the complexity of exports [14, 15]. Hummels et al. [16] measured vertical specialization level and growth and defined vertical specialization with import intermediate input as a key factor when producing export products. However, their calculation method controlled strict assumptions. Daudin et al. [17] redistributed the trade flow to the original input-production industries and countries and proposed a new standard for measuring value-added trade in international trade. Koopman et al. [18] assumed that there is no two-way trade of intermediate goods, normalized the calculated indicators in a linear combination, decomposed the export trade of a single decision-making unit into four parts, and proposed the KWW model, which has been widely used by scholars. In terms of the factors influencing the division of labor position in the GVC, the technological level and endowment structure of factors are crucial for a country to participate in the division of labor in the GVC [19]. According to the competitive advantage staged development model, the driving force of position improvement in the GVC is the transformation from simple factor capital to innovative capital. At the same time, the GVC position will also affect the international flow of technological innovation. There is a causal relationship between these variables [20]. Based on an empirical study of China and Mexico, Gallagher and Shafaeddin [21] concluded that technological upgrading and independent innovation are important factors in promoting a country's deep participation in the division of labor in the GVC. In addition, academics have studied the impact of infrastructure on the GVC position. The infrastructure construction process is often accompanied by the redistribution of many resource factors, such as capital, talent, and technology [22–25]. Infrastructure connectivity can promote trade and investment facilitation and reduce the cost of factor flow [26–28]. Some scholars believe that intellectual property protection is an important factor that affects the innovation capacity of service industries and improving the level of intellectual property protection is conducive to the technological innovation of service industries [29, 30]. By establishing a multicountry and multistage GVC competition model, many studies have proposed that in the division of the labor process in the GVC, improving the technological level and reducing the factor cost are the main ways to promote the upgrading of a country's GVC [31, 32]. There is an inverted *U*-shaped relationship between R&D subsidies and the GVC position, and Internet penetration can weaken the inverted *U*-shaped relationship [33]. Furthermore, the study shows that foreign direct investment (FDI) is an important factor affecting the participation of the division of labor in the GVC of the digital services industry. FDI can improve the technological level of capital inflow to countries through the technology spillover effect, deepen a country's participation in the GVC, and effectively improve a country's division of labor position of a country in the GVC [34, 35].

Based on the statement above, AI technology has great potential for application to cultural industries. Scholars have conducted many studies on how AI can promote the development of cultural industries, but there are at least two deficiencies in existing research: (1) Few studies examine the impact of AI on the development of cultural industries, and only at the technical level; there is a lack of research on GVC position and quantitative analysis of the impact of AI on cultural industries from the trade level. (2) There is a lack of research on how AI technology has a heterogeneous impact on the development of cultural industries in high-income and low- and middle-income countries. Based on the theory of GVC and the panel data of 56 countries and regions from 2010 to 2018, this study empirically analyzes the impact of AI on improving the GVC position of cultural industries in each country. For countries at different levels of economic development, this effect shows heterogeneity. Heterogeneity analysis is also carried out for different stages of economic development. These research results have theoretical value and practical significance for the development of AI and the formulation of relevant policies, the high-quality development of cultural industries, and path selection for promoting the GVC position and provide a reference for upgrading the GVC of cultural industries.

The rest of the article is organized as follows: Section 3 describes the research methods. The double fixed effects regression model is introduced to verify the impact of AI on the GVC position of cultural industries. Based on the benchmark regression analysis, endogeneity, and robustness test, the influence mechanisms of AI on the promotion of the GVC position of cultural industries are examined in Section 4. This step is followed by analyzing the influence of heterogeneity based on different stages of economic development, and the results of models are discussed. The conclusions and some practical suggestions for upgrading the GVC of cultural industries are outlined in Section 6.

## 3. Research Methods

### 3.1. Model Setup

Most previous studies have used an ordinary least squares (OLS) model that has only considered the explanatory factors of the division of labor position in the GVC of industries with cross-sectional data but has ignored some variables in the actual development and the disturbance to the GVC position of industries caused by individual and time changes. In practice, many factors affect the GVC position of cultural industries, such as international emergencies. These factors change with time but not with countries and regions. Therefore, the time fixed effect is included in the model to ensure the accuracy of the analysis [36]. At the same time, different countries and regions show differences in unobservable factors that do not change over time, such as geographical location and consumption habits. Therefore, this study adds an individual fixed effect to the model [36]. To verify the impact of AI on the GVC position of cultural industries, this study constructs a double fixed effects regression model, and the econometric model is as follows:

(1) $$\begin{array}{c} {\text{GVC}}_{\text{it}}=\beta_{0}+\beta_{1}{\text{AI}}_{\text{it}}+\beta Z_{\text{it}}+\theta_{t}+\gamma_{i}+\varepsilon_{\text{it}}, \end{array}$$

where *i* is a country or region, *t* stands for year, GVC_it_ is the explained variable, representing the GVC position of cultural industries in country (region) *i* in year *t*, AI_it_ is the explanatory variable, representing the level of AI development of country (region) *i* in year *t*, *β* is the parameter to be estimated, *Z*_it_ indicates other control variables affecting the cultural industries, *ε*_it_ is a random disturbance term, *θ*_*t*_ is the time fixed effect, and *γ*_*i*_ is an individual fixed effect.

### 3.2. Description of Variables

#### 3.2.1. Explained Variable

The explained variable in this study is the GVC position index of cultural industries, which represents the position of a country or region's cultural industries in the GVC. The GVC position can reflect the degree to which cultural industries participate the GVC production activities of a country (region). Koopman et al. [37] proposed a method to calculate the GVC position using value-added trade to measure the position of the producers of the industries in the GVC. Wang et al. [38] calculated the GVC position index based on forward linkage and backward linkage, which is considered highly representative in academia. Following the method used by Wang et al., the production length of GVC based on forward and backward linkages can be expressed as follows:

(2) $$\begin{array}{c} \text{PLv\_GVC}=\text{PLvd\_GVC}+\text{PLvi\_GVC}=\frac{\text{Xv\_GVC}}{\text{V\_GVC}}\text{,} \end{array}$$

(3) $$\begin{array}{c} \text{PLy\_GVC}=\text{PLyd\_GVC}+\text{PLyi\_GVC}=\frac{\text{Xy\_GVC}}{\text{Y\_GVC}}\text{,} \end{array}$$

where PLvd_GVC represents the domestic length of the forward linkage GVC, PLvi_GVC represents the international length of the forward linkage GVC, Xv_GVC represents the total output caused by the export of intermediate goods, V_GVC represents all exports of intermediate goods, PLyd_GVC represents the domestic length of backward linkage GVC, PLyi_GVC represents the international length of backward linkage GVC, Xy_GVC represents the total output caused by initial input, Y_GVC represents the total output of production activities participating in GVC, PLv_GVC indicates the production length of the forward linkage GVC, and PLy_GVC indicates the production length of the backward linkage GVC.

The position of cultural industries in GVC production is expressed by using the ratio of the length of the forward linkage value chain and the length of the backward linkage value chain.

(4) $$\begin{array}{c} \text{GVCPs}=\frac{\text{PLv\_GVC}}{\text{PLy\_GVC}}\text{,} \end{array}$$

where GVCPs represents the GVC position index of a country's or region's cultural industries. The larger the index is, the higher the position of the country's cultural industries in the GVC is.

#### 3.2.2. Explanatory Variable

Currently, in terms of AI measurement, the measurement angle is still relatively singular. AI patent data are often taken as a proxy variable, reflecting the development characteristics and trends of the AI industry [39]. To analyze the influence of AI on cultural industries in countries (regions), this study follows the method of Agrawal et al. [40] and selects the ratio of the number of robots in countries (regions) to the number of jobs in service industries as the proxy variable of the level of AI development. The term “robot” in this study is defined by the International Organization for Standardization (ISO) as an automatic, programmable, multifunctional, and fixed or mobile industrial device consisting of three or more rotating shafts. Given the comparability and availability of data at the international level, the robot stock of countries and regions reported by the International Federation of Robotics (IFR) and the employment number of countries and regions in service industries according to the International Labor Organization are selected to measure the development level of AI.

#### 3.2.3. Control Variables

The development level of AI is one of the complex and diverse factors influencing the position of cultural industries in the GVC, the development level of AI is only one of them. Control variables are designed based on the existing research. The selected control variables include human capital (HC), intellectual property protection (IPP), infrastructure quality (Infra), level of economic development (GDPP), and foreign direct investment (FDI).

*(1) Human Capital (HC)*. As the level and quality of the elements in the GVC division system are important factors determining the position of the division of labor, human capital has a certain influence on the position of cultural industries in the GVC. This study uses the World Bank database of higher education enrolment rates to measure the level of human capital. The indicator calculates the number of university students as a percentage of the total postsecondary school-age population.

*(2) Intellectual Property Protection (IPP)*. The intellectual property protection index of the Global Competitiveness Report of the World Economic Forum is adopted to measure the level of intellectual property protection of a country (region). The index ranges from 1 to 7, with a higher score indicating a higher level of intellectual property protection in an economy.

*(3) Quality of Infrastructure (Infra)*. This study uses the global infrastructure quality index of countries (regions) in the Global Competitiveness Report of the World Economic Forum to measure infrastructure quality. The index ranges from 1 to 7, with a higher score indicating that an economy has a more developed infrastructure.

*(4) Economic Development Level (GDPP)*. The level of economic development is measured by GDP per capita from the World Bank database.

*(5) Foreign direct investment (FDI)*. The proportion of net FDI inflow in GDP from the World Bank database is used to measure the level of FDI utilization in a country or region.

### 3.3. Sample Selection and Data Sources

The original data on the GVC of cultural industries used in the econometric model in this study come from the OECD TiVA database mainly because it has the same statistical caliber and high authority at the country level. The database links the international input-output tables of 66 economies (countries and regions) and analyzes in detail all transactions between economies and industries in 45 industries from a global perspective. Among them, the statistical scope of cultural industries includes publishing, audiovisual, and broadcasting activities. Therefore, this study uses the UIBE-GVC database to calculate the GVC position index of cultural industries. In terms of the explanatory variable, AI development level data come from the IFR and the International Labor Organization. The stock of robots is one of the more commonly used measures of AI, and the IFR is the world's foremost authority on robot data. This study focuses on the aspects of information dissemination and services of cultural industries, excluding the production, sales, and leasing of telecommunications products. Then, the OECD TiVA database is matched with countries and regions in the IFR database and the World Bank database according to the 4th edition of the United Nations International Standard Industry Classification (ISIC Rev 4.0) and excludes Costa Rica, Luxembourg, the Slovak Republic, Brunei Darussalam, Cambodia, Cyprus, Kazakhstan, the Lao People's Democratic Republic, Myanmar, and Chinese Taipei. These 10 countries or regions do not have subsectors in the database. In terms of control variables, IPP and Infra are from the World Bank database, while HC, GDPP, and FDI are from the World Economic Forum Global Competitiveness Report. GDPP and FDI are calculated according to the current US$. To reduce heteroscedasticity and multicollinearity among the data, the natural logarithm of HC, IPP, Infra, and GDPP is adopted in the model construction. Based on data availability and consistency, this study selected cultural industry data from the remaining 56 countries or regions in the OECD TiVA database from 2010 to 2018 to construct panel data. The descriptive statistics of the sample data are shown in Table 1 under the condition that consistency of statistical caliber follows and a few missing data are interpolated.

## 4. Empirical Results and Analysis

### 4.1. Benchmark Regression Analysis

In this study, considering the possible heteroscedasticity of the model, the Hausman test shows that the sample data have individual fixed effects and time fixed effects. Therefore, the double fixed effects regression model calculated by OLS is used to empirically test model (1). EViews 12 is used for calculating the results of model estimation. The benchmark regression results shown in Table 2 show the impact of AI development on the GVC position of cultural industries. Column (1) is the regression result of individual and time effects considering only the core variable AI; column (2) is the regression result of controlling the individual fixed effects of the model considering all the control variables included in the econometric model; and column (3) is the result of the double fixed effects regression model. The explanatory variable coefficients of columns (1), (2), and (3) in Table 2 are close, indicating that the results of the model estimation are relatively robust. The results of the double fixed effects model show that the regression coefficient between AI and GVCPs is 0.0047, and it is significant at the 1% level, indicating that AI development has a positive effect on the division of labor position of a country (region) in the GVC. In terms of the value of the regression coefficient, AI has a slightly weak positive impact on the GVC position of cultural industries. This situation is caused mainly by the fact that, AI is still in the weak development stage in cultural industries, that is, data intelligence. There is still much scope for developing the technology itself and its application fields, and the promotional role of cultural industries in the GVC has not been fully demonstrated.

### 4.2. Endogeneity and Robustness Tests

#### 4.2.1. Endogeneity Test

The development of cultural industries in a country (region) has a limited impact on the development of AI in that area. However, to effectively solve the possible endogeneity problem caused by two-way causality in the model, this study uses EViews 12 to replace the original explanatory variable with a lagged explanatory variable with one lag period for the endogenous test and rerun the OLS regression, which can avoid inverse relationships. The regression results of instrumental variables reported in columns (1) to (3) of Table 3 show that AI plays a significant role in improving the GVC position of cultural industries at the 1% significance level, which is consistent with the previous results, indicating the validity of the research results.

#### 4.2.2. Robustness Test

To further ensure the effectiveness of the impact of AI on the GVC position of cultural industries, this study uses EViews 12 to conduct a robustness test by changing the measure of the explanatory variable. At present, few studies conduct a quantitative analysis of AI, and there are limited references for the selection of alternative variables. This study changes the explanatory variable from AI to the citations of the AI academic achievements (AI_C) to measure AI development. AI_C refers to the citations of the AI topic category in the core collection database of Web of Science and the Scimago Journal & Country Rank (SJR) database. In addition, the logarithm of AI_C is taken to repeat the OLS regression. The regression results from columns (4) to (6) in Table 3 are basically consistent with the benchmark regression results in Table 2 in terms of the direction, magnitude, and significance level of the explanatory variable and control variables. These results indicate that the regression results in this study are robust.

### 4.3. Mechanism Test

The regression analysis has shown that the development of AI can improve the GVC position of cultural industries, but the mechanisms by which this improvement occurs need to be further tested. This study will examine the influence mechanisms of AI on the promotion of the GVC position of cultural industries in terms of technological innovation and the industrial structure.

#### 4.3.1. Technological Innovation Effect

Technological iteration and application popularization will not only directly enhance cultural productivity, stimulate the tertiary industry, and further optimize the economic structure but also promote the innovation behavior of cultural enterprises. With the continuous application of AI, barriers between traditional cultural products and digital technology are continually being eliminated. The combination of the two is conducive to improving cultural consumption, providing favorable conditions for innovating the production mode of cultural products, and achieving the high-quality development of cultural industries. To analyze the influence of AI on the GVC position of cultural industries through the effect of technological innovation, the ratio of R&D expenditure to GDP in the World Bank database is adopted as the index to measure technological innovation (RD). Based on model (1), the mediating effect models (5) and (6) are constructed.

(5) $$\begin{array}{c} {\text{RD}}_{\text{it}}=\beta_{0}+\beta_{1}{\text{AI}}_{\text{it}}+\beta Z_{\text{it}}+\theta_{t}+\gamma_{i}+\varepsilon_{\text{it}}, \end{array}$$

(6) $$\begin{array}{c} {\text{GVC}}_{\text{it}}=\beta_{0}+\beta_{1}{\text{AI}}_{\text{it}}+\beta_{2}{\text{RD}}_{\text{it}}+\beta Z_{\text{it}}+\theta_{i}+\gamma_{i}+\varepsilon_{\text{it}}. \end{array}$$

Table 4 lists the results of the effect of the mediating variable RD on the relationship between AI and the GVC position of cultural industries. Table 4 shows that the AI coefficients of all models are significantly positive based on a comparison of the results of the fixed effects regression model with or without the inclusion of RD, the lagged explanatory variable regression model, and the replacement explanatory variable regression model. Column (1) is listed as the regression result of the benchmark. Column (2) reports the effect of AI on the mediating variable RD. The influence coefficient between AI and RD is 0.0520, which is significant at the 1% level, indicating that the development of AI has effectively promoted the level of technological innovation of a country (region). According to the regression results in column (3), AI has a significantly positive impact on the GVC position of cultural industries, while technological innovation has a smaller impact on the GVC position of cultural industries. Columns (4) and (5) are listed as the results of endogeneity test and robustness test, respectively. Moreover, technological innovation has a partial mediating effect, and the role of AI in improving the GVC position of cultural industries by improving the level of technological innovation needs to be further encouraged. Most cultural enterprises are in the growth stage, and their production mode, management mode, and business form urgently need to adapt to the era of AI to achieve effective transformation. Therefore, AI will play an increasingly important role in stimulating innovation, improving the added value of products, and promoting industrial innovation.

#### 4.3.2. Industrial Structure Effect

AI is a general technology with new infrastructure, and its application prospect is quite different in different industries, which will cause a change in the industrial structure. To analyze the influence of AI on the GVC position of cultural industries through the industrial structure effect, the ratio of the added value of service industries to GDP in the OECD TiVA database is adopted as an indicator to measure industry structure (Industry). Based on model (1), mediating effect models (7) and (8) are constructed.

(7) $$\begin{array}{c} {\text{Industry}}_{\text{it}}=\beta_{0}+\beta_{1}{\text{AI}}_{\text{it}}+\beta Z_{\text{it}}+\theta_{t}+\gamma_{i}+\varepsilon_{\text{it}}, \end{array}$$

(8) $$\begin{array}{c} {\text{GVC}}_{\text{it}}=\beta_{0}+\beta_{1}{\text{AI}}_{\text{it}}+\beta_{2}{\text{Industry}}_{\text{it}}+\beta Z_{\text{it}}+\theta_{t}+\gamma_{i}+\varepsilon_{\text{it}}. \end{array}$$

Table 5 lists the results of the effect of the mediating variable Industry on the relationship between AI and the GVC position of cultural industries. Table 5 shows that the AI coefficients in all models are significantly positive based on a comparison of the results of the fixed effects regression model with or without the inclusion of Industry, the lagged explanatory variable regression model, and the replacement explanatory variable regression model. Column (1) is listed as the regression result of the benchmark. Column (2) reports the effect of AI on the intermediary variable Industry. The impact of AI on the industrial structure is significantly positive, indicating that AI effectively improves the industrial structure of a country (region). Based on the regression results of column (3), the influence coefficient between Industry and GVCPs is 0.0578, which is significant at the 1% level, and the influence of AI on the GVC position of cultural industries is significantly positive. Columns (4) and (5) are listed as the results of endogeneity test and robustness test, respectively. The results show that AI has a mediating effect on improving the division of labor position of cultural industries in the GVC through the industrial structure, that is the development of AI will indeed improve the division of labor position in the GVC of cultural industries by promoting the upgrades of the industrial structure.

## 5. Further Analysis Based on the Stages of Economic Development

According to the analysis above, the discussion of AI and the GVC position of cultural industries is conducted on a global scale. However, the international environment is very complex, and the income level of a country (region) affects the situation of the GVC position of cultural industries in the country (region). Additionally, Agrawal et al. found that AI has heterogeneous impacts on the labor forces in countries with different income levels, industries, and genders. To analyze the potential heterogeneity effect, 56 countries (regions) in the sample are divided into two subsamples, namely high-income countries (regions) and low- and middle-income countries (regions). According to the classification standard of the World Bank, the former corresponds to “high-income countries (regions),” while the latter includes three categories: “upper middle-income countries (regions),” “lower middle-income countries (regions),” and “low income countries (regions).”

The regression results based on the above sample classification are shown in Table 6. After the addition of control variables, in the sample of high-income countries (regions), AI has a significant positive role in improving the GVC position of cultural industries. For low- and middle-income countries (regions), this effect is not significant. This difference may be due to two reasons: (1) High-income countries (regions) are the main drivers of the development and application of AI. In the process of adjusting the GVC, high-income countries (regions) accumulate technological advantages to gain control over creative design, high-end research and development, and branding and marketing of high-technology and high value-added products in the global culture industry chain. To maintain a dominant position in the value chain of the global cultural industry, high-income countries (regions) have set up links with high barriers to entry. Then, as high-income countries invest their higher incomes in technological innovation, creative research, and the development of cultural products, their high value-added competitive advantages become more obvious, and the gap between them and low- and middle-income countries in the GVC widens. (2) In contrast, due to the constraints of policies, talent, resources, technology, and the market environment in some low- and middle-income countries (regions), there is a large gap in the research and development of emerging technologies in cultural industries with high-income countries (regions), and there are great differences in the technological level and the endowment conditions of the factors. These differences suggest that different countries (regions) will also have different attitudes towards AI technology. In some countries, the application of AI technology in cultural industries is weak due to the incompatibility of AI technology with the factor endowment structure, an incomplete cultural industry system, factor mismatches, structural contradictions, and imperfect governance mechanisms, which are not conducive to improving the GVC position of cultural industries in these countries (regions).

## 6. Conclusions

With the rapid development of AI technology, the upgrading of cultural industries has ushered in a new digital era, creating many new forms of industries. The transformation of cultural industries by AI has entered a new stage and is constantly promoting the reconstruction of the GVC. First, this study uses cross-border panel data to measure the level of AI development with respect to robot stock and constructs a double fixed effects regression model to empirically analyze the impact of AI on improving the GVC position of cultural industries. Second, to overcome the possible endogeneity problem of the model, the endogeneity test of the benchmark regression results is carried out using a lagged explanatory variable with one lag period as the instrumental variable, and the robustness test is carried out by changing the measure of the explanatory variable using the replacement explanatory variable method. In addition, the study examines the influence mechanisms of AI on the promotion of the GVC position of cultural industries in terms of technological innovation and industrial structure. Finally, the heterogeneous effect of AI on the GVC position of cultural industries in different stages of economic development is further analyzed. The results show that (1) AI has a significant impact on improving the GVC position of cultural industries. (2) The mechanism test confirmed that AI has a mediating effect on improving the division of labor position in the GVC of cultural industries through the industrial structure. The role of AI in improving the GVC position of cultural industries by improving the level of technological innovation needs to be further encouraged. (3) The level of AI development has a heterogeneous impact on cultural industries in countries or regions with different income levels. AI has a significant positive role in improving the GVC position of cultural industries in high-income countries (regions), while it has no significant impact on low- and middle-income countries (regions). Although this article examines the influence mechanisms of AI on the promotion of the GVC position of cultural industries in terms of technological innovation and the industrial structure, it does not carry out in-depth discussion on how its impact mechanisms work. Future researchers can conduct more in-depth analyses of the aspect.

From the perspective of the development of the world's cultural industries, large-scale and artificial intelligence represent inevitable trends in future technologically based development, and the deep integration of cultural industries and AI is of great significance. Therefore, this study provides the following recommendations:

1. Vigorously develop AI technology related to cultural industries. Technological innovation, as an endogenous driving force, is the core element in enhancing the technological innovation ability of cultural industries. Therefore, in the era of AI, scientific and technological innovation should be accelerated, the production productivity of cultural products should be improved, cultural formats and product forms should be innovated, the internal restructuring of cultural industries should be promoted, and a cultural production system with international competitiveness should be constructed.
2. As an important way to improve the international competitiveness of cultural industries, the application of AI technology should be vigorously promoted. It is necessary to fully recognize the importance of the deep integration strategy of AI and cultural industries and to take advantage of the opportunities that AI offers the cultural industries. More importantly, AI provides a new advantage in the international competition of cultural industries to promote industrial transformation, innovation upgrading, and applications of AI in the field of cultural industries.
3. From the perspective of resource allocation, in the process of iteration and integration of new and old cultural industries, it is necessary to make a rational use of resources from the policy environment, production factor resources, and market factor resources, to better drive the upgrading of cultural industries by optimizing resource allocation.
4. A high-quality institutional environment is the key to the efficient and orderly operation of cultural industries. Optimizing the policy environment of cultural industries and further refining the industrial system can guarantee the position of cultural industries in the global cultural market competition and help realize the high-quality development of cultural industries. In addition, it is necessary to focus on cultivating the talents of high-quality cultural industries, encourage all types of cultural enterprises to fully exploit their strengths, deeply participate in the division of labor and cooperation among international cultural industries, and comprehensively improve their GVC position.

## Figures and Tables

**Table 1:** Descriptive statistics of sample data.

Variable category	Variable name	Variable description	*N*	Mean	Std	Min	Max
Explained variable	GVCPs	GVC position index	504	1.0075	0.1083	0.6983	1.3505

Explanatory variables	AI	Artificial intelligence	504	1.3678	2.0939	0.0003	16.0343
	HC	Human capital	504	4.1032	0.4041	2.6788	4.9618
	IPP	Intellectual property protection	504	1.4986	0.2422	0.8478	1.8841

Control variables	Infra	Quality of infrastructure	504	1.5980	0.1821	1.0722	1.9132
	GDPP	Economic development level	504	9.7817	1.0452	7.0878	11.5416
	FDI	Foreign direct investment	504	4.9016	11.1519	−40.0811	102.3137

**Table 2:** Regression results of the benchmark.

Variables	GVCPs		
	(1)	(2)	(3)
AI	0.0048^*∗∗∗*^ (2.5838)	0.0037^*∗∗*^ (2.1206)	0.0047^*∗∗*^ (2.5067)
HC		0.0364^*∗∗∗*^ (2.8733)	0.0390^*∗∗∗*^ (2.8737)
IPP		0.0291^*∗*^ (1.8274)	0.0243 (1.1345)
Infra		−0.0191 (−0.8994)	0.0143 (0.4831)
GDPP		0.0056 (0.5167)	0.0142 (1.1622)
FDI		0.0001 (0.0846)	−0.0001 (−0.2666)
Constants	1.0010^*∗∗∗*^ (360.3240)	0.7850^*∗∗∗*^ (7.5368)	0.6436^*∗∗∗*^ (5.3180)
Individual fixed effect	Yes	Yes	Yes
Time fixed effect	Yes	No	Yes
*R*-squared	0.9447	0.9553	0.9560
*N*	504	504	504

Robust *t*-statistics in parentheses, ^*∗∗∗*^*p* < 0.01, ^*∗∗*^*p* < 0.05, ^*∗*^*p* < 0.1.

**Table 3:** Endogeneity and robustness tests.

Variables	GVCPs					
	(1)	(2)	(3)	(4)	(5)	(6)
L. AI	0.0056^*∗∗∗*^ (2.4843)	0.0040^*∗*^ (1.9175)	0.0054^*∗∗*^ (2.4337)			
AI_C				0.0038^*∗∗∗*^ (3.0002)	0.0035^*∗∗∗*^ (2.7348)	0.0036^*∗∗∗*^ (2.7839)
HC		0.0476^*∗∗∗*^ (3.3213)	0.0515^*∗∗∗*^ (3.3483)		0.0409^*∗∗∗*^ (3.3193)	0.0413^*∗∗∗*^ (3.0634)
IPP		0.0370^*∗∗*^ (2.3013)	0.0366^*∗*^ (1.6759)		0.0254 (1.5833)	0.0136 (0.6339)
Infra		−0.0222 (−1.0783)	0.0141 (0.4773)		−0.0185 (−0.8764)	0.0045 (0.1515)
GDPP		0.0127 (1.1036)	0.0172 (1.3639)		0.0059 (0.5418)	0.0159 (1.3031)
FDI		0.0002 (1.0684)	0.0001 (0.6267)		−0.0001 (−0.0645)	−0.0001 (−0.3152)
Constants	1.0006^*∗∗∗*^ (320.6268)	0.6616^*∗∗∗*^ (5.6632)	0.5425^*∗∗∗*^ (4.1987)	0.9761^*∗∗∗*^ (92.5578)	0.7453^*∗∗∗*^ (7.2430)	0.6263^*∗∗∗*^ (5.1775)
Individual fixed effect	Yes	Yes	Yes	Yes	Yes	Yes
Time fixed effect	Yes	No	Yes	Yes	No	Yes
*R*-squared	0.9610	0.9624	0.9630	0.9547	0.9556	0.9562
*N*	448	448	448	504	504	504

Robust *t*-statistics in parentheses, ^*∗∗∗*^*p* < 0.01, ^*∗∗*^*p* < 0.05, ^*∗*^*p* < 0.1.

**Table 4:** Mechanism test (technical innovation).

Variables	GVCPs	RD	GVCPs	GVCPs	GVCPs
	(1)	(2)	(3)	(4)	(5)
AI	0.0047^*∗∗*^ (2.5067)	0.0520^*∗∗∗*^ (4.4644)	0.0057^*∗∗∗*^ (2.9772)		
L.AI				0.0063^*∗∗∗*^ (2.8060)	
AI_C					0.0035^*∗∗∗*^ (2.7272)
RD			−0.0187^*∗∗*^ (−2.4443)	−0.0199^*∗∗*^ (−2.4519)	−0.0132^*∗*^ (−1.7620)
Control variables	Yes	Yes	Yes	Yes	Yes
Constants	0.6436^*∗∗∗*^ (5.3180)	0.4041 (0.5254)	0.6511^*∗∗∗*^ (5.4094)	0.5419^*∗∗∗*^ (4.2217)	0.6319^*∗∗∗*^ (5.2346)
Individual fixed effect	Yes	Yes	Yes	Yes	Yes
Time fixed effect	Yes	Yes	Yes	Yes	Yes
*R*-squared	0.9560	0.9814	0.9566	0.9636	0.9565
*N*	504	504	504	448	504

Robust *t*-statistics in parentheses, ^*∗∗∗*^*p* < 0.01, ^*∗∗*^*p* < 0.05, ^*∗*^*p* < 0.1.

**Table 5:** Mechanism test (industrial structure).

Variables	GVCPs	Industry	GVCPs	GVCPs	GVCPs
	(1)	(2)	(3)	(4)	(5)
AI	0.0047^*∗∗*^ (2.5067)	0.0138^*∗*^ (1.6493)	0.0039^*∗∗*^ (2.1440)		
L.AI				0.0048^*∗∗*^ (2.2259)	
AI_C					0.0032^*∗∗∗*^ (2.5934)
Industry			0.0578^*∗∗∗*^ (5.5756)	0.0587^*∗∗∗*^ (5.2658)	0.0582^*∗∗∗*^ (5.6388)
Control variables	Yes	Yes	Yes	Yes	Yes
Constants	0.6436^*∗∗∗*^ (5.3180)	−2.1503^*∗∗∗*^ (−3.9686)	0.7679^*∗∗∗*^ (6.4455)	0.6879^*∗∗∗*^ (5.3789)	0.7532^*∗∗∗*^ (6.3277)
Individual fixed effect	Yes	Yes	Yes	Yes	Yes
Time fixed effect	Yes	Yes	Yes	Yes	Yes
R-squared	0.9560	0.9734	0.9590	0.9656	0.9592
N	504	504	504	448	504

Robust *t*-statistics in parentheses, ^*∗∗∗*^*p* < 0.01, ^*∗∗*^*p* < 0.05, ^*∗*^*p* < 0.1.

**Table 6:** Heterogeneous effect of AI on the GVC position of cultural industries.

Variables	GVCPs					
	High-income countries (regions)			Low- and middle-income countries (regions)		
	(1)	(2)	(3)	(4)	(5)	(6)
AI	0.0056^*∗∗∗*^ (2.92)	0.0050^*∗∗∗*^ (2.5511)		0.0169 (1.3956)	0.0083 (0.5749)	
L. AI			0.0062^*∗∗∗*^ (2.5468)			−0.0211 (−1.4127)
HC		0.0444^*∗∗*^ (2.1379)	0.0477^*∗∗*^ (1.9477)		0.0140 (0.6716)	0.0458^*∗∗*^ (2.1709)
IPP		−0.0073 (−0.1875)	0.0183 (0.4385)		0.0030 (0.0974)	0.0119 (0.4297)
Infra		0.0443 (1.0165)	0.0627 (1.3687)		0.0108 (0.1995)	−0.0278 (−0.5724)
GDPP		0.0120 (0.0789)	0.0143 (0.7867)		0.0218 (1.0326)	0.0356^*∗*^ (1.8302)
FDI		−0.0001 (−0.1269)	0.0001 (0.7793)		0.0001 (0.0316)	0.0022 (0.9120)
Constants	0.9997^*∗∗∗*^ (255.9682)	0.0628^*∗∗∗*^ (3.2828)	0.5136^*∗∗*^ (2.4173)	0.9968^*∗∗∗*^ (242.8421)	0.7318^*∗∗∗*^ (4.1766)	0.5309^*∗∗∗*^ (3.3079)
Individual fixed effect	Yes	Yes	Yes	Yes	Yes	Yes
Time fixed effect	Yes	Yes	Yes	Yes	Yes	Yes
*R*-squared	0.9350	0.9365	0.9431	0.9738	0.9743	0.9827
*N*	333	333	296	171	171	152

Robust *t*-statistics in parentheses, ^*∗∗∗*^*p* < 0.01, ^*∗∗*^*p* < 0.05, ^*∗*^*p* < 0.1.

## Data Availability

The data that support the findings of this study are included within the article.

## References

[1] Moran M. (2008). Three laws of robotics and surgery. *Journal of Endourology*.

[2] Zhang H., Cui Y. (2019). A model combining a bayesian network with a modified genetic algorithm for green supplier selection. *Simulation-Transactions of the Society for Modeling and Simulation International*.

[3] Zhang H. P. (2019). Optimization of remanufacturing production scheduling considering uncertain factors. *International Journal of Simulation Modelling*.

[4] Xu W., Sun H. Y., Awaga A. L., Yan Y., Cui Y. J. (2022). Optimization approaches for solving production scheduling problem: a brief overview and a case study for hybrid flow shop using genetic algorithms. *Advances in Production Engineering & Management*.

[5] Venkatesan D., Kannan K., Saravanan R. (2009). A genetic algorithm-based artificial neural network model for the optimization of machining processes. *Neural Computing & Applications*.

[6] Ciurea C., Pocatilu L., Filip F. G. (2020). Using modern information and communication technologies to support the access to cultural values. *Journal of System and Management Sciences*.

[7] Rahwan I., Cebrian M., Obradovich N. (2019). Machine behaviour. *Nature*.

[8] Goel P., Kaushik N., Sivathanu B., Pillai R., Vikas J. (2022). Consumers’ adoption of artificial intelligence and robotics in hospitality and tourism sector: literature review and future research agenda. *Tourism Review*.

[9] Gajsek B., Marolt J., Rupnik B., Lerher T., Sternad M. (2019). Using maturity model and discrete-event simulation for industry 4.0 implementation. *International Journal of Simulation Modelling*.

[10] Srinivasan S. M., Shah P., Surendra S. (2021). An approach to enhance business intelligence and operations by sentimental analysis. *Journal of System and Management Sciences*.

[11] Shahzad F., Xiu GY., Shahbaz M. (2017). Organizational culture and innovation performance in Pakistan’s software industry. *Technology in Society*.

[12] Naveed K., Watanabe C., Neittaanmäki P. (2017). Co-evolution between streaming and live music leads a way to the sustainable growth of music industry-lessons from the US experiences. *Technology in Society*.

[13] Acemoglu D., Restrepo P. (2018). The race between man and machine: implications of technology for growth, factor shares, and employment. *The American Economic Review*.

[14] Antràs P., Chor D., Fally T., Hillberry R. (2012). Measuring the upstreamness of production and trade flows. *The American Economic Review*.

[15] Hausmann R., Hwang J., Rodrik D. (2007). What you export matters. *Journal of Economic Growth*.

[16] Hummels D., Ishii J., Yi K. M. (2001). The nature and growth of vertical specialization in world trade. *Journal of International Economics*.

[17] Daudin G., Rifflart C., Schweisguth D. (2011). Who produces for whom in the world economy?. *Canadian Journal of Economics*.

[18] Koopman R., Wang Z., Wei S. J. (2012). Estimating domestic content in exports when processing trade is pervasive. *Journal of Development Economics*.

[19] Grossman G. M., Rossi-Hansberger E. (2012). Task trade between similar countries. *Econometrica*.

[20] Caselli F., Coleman W. J. (2006). The world technology frontier. *The American Economic Review*.

[21] Gallagher K. P., Shafaeddin M. (2010). Policies for industrial learning in China and Mexico. *Technology in Society*.

[22] Banerjee A. E., Duflo E., Qian N. (2020). On the road: access to transportation infrastructure and economic growth in China. *Journal of Development Economics*.

[23] Zhang H., Wang M. K., Tang M. J., Yang H. X. (2018). The reliability measures model of multilayer urban distribution network. *Soft Computing*.

[24] Ju S. W., Park Y. S. (2022). Public design method based on smart service system technology: centered on the cases of bus stops in Korea and China. *Journal of Logistics, Informatics and Service Science*.

[25] Zhang L., Yan Y., Xu W., Sun J., Zhang Y. Y. (2022). Carbon emission calculation and influencing factor analysis based on industrial big data in the “double carbon” Era. *Computational Intelligence and Neuroscience*.

[26] Gorg H., Greenaway D. (2004). Much ado about nothing? do domestic firms really benefit from foreign direct investment?. *The World Bank Research Observer*.

[27] Zhang H., Tang L., Yang C., Lan S. L. (2019). Locating electric vehicle charging stations with service capacity using the improved whale optimization algorithm. *Advanced Engineering Informatics*.

[28] Jang J., Kyun S. (2022). An innovative career management platform empowered by ai, big data, and blockchain technologies: focusing on female engineers. *Journal of Logistics, Informatics and Service Science*.

[29] Miles I., Andersen B., Howells J., Boden M. (2000). Service production and intellectual property. *International Journal of Technology Management*.

[30] Dey M., Houseman S. N., Polivka A. E. (2012). Manufacturers’ outsourcing to staffing services. *ILR Review*.

[31] Lee E., Yi K. M. (2018). Global value chains and inequality with endogenous labor supply. *Journal of International Economics*.

[32] Antràs P., Gortari A. (2020). On the geography of global value chains. *Econometrica*.

[33] Konings J. (2001). The effects of foreign direct investment on domestic firms: evidence from firm level panel data in emerging economies. *The Economics of Transition*.

[34] Thorbecke W. (2018). Investigating ASEAN’s electronic and labor-intensive exports. *Journal of Asian Economics*.

[35] Qian F. R., Yuan X. Y. (2022). R&D subsidies, internet penetration and global value chain position. *R & D Management*.

[36] Abadie A., Gardeazabal J. (2003). The economic costs of conflict: a case study of the Basque country. *The American Economic Review*.

[37] Koopman R., Wang Z., Wei S. J. (2014). Tracing value-added and double counting in gross exports. *The American Economic Review*.

[38] Wang Z., Wei S. J., Yu X. (2017). *Characterizing Global Value Chains: Production Length and Upstreamness*.

[39] Fujii H., Managi S. (2018). Trends and priority shifts in artificial intelligence technology invention: a global patent analysis. *Economic Analysis and Policy*.

[40] Agrawal A., Gans J. S., Goldfarb A. (2019). Artificial intelligence: the ambiguous labor market impact of automating prediction. *The Journal of Economic Perspectives*.

